RETRACTED

# Long noncoding RNA UBA6-AS1 inhibits the malignancy of ovarian cancer cells via suppressing the decay of UBA6 mRNA

**DOI:** 10.1080/21655979.2021.2011640

**Published:** 2021-12-24

**Authors:** Yaogang Wang, Zhigao Chen

**Affiliations:** Department of Gynaecology and Obstetrics, Hanchuan People’s Hospital, Hanchuan, Hubei Province, China

**Keywords:** M^6^a modification, RBM15, RNA stability, IGF2BP1

## Abstract

Ovarian cancer (OC) is one of the most common cancer in women worldwide. A recent study reported that long noncoding RNA (lncRNA) Ubiquitin like modifier activating enzyme 6 antisense RNA 1 (UBA6-AS1) is significantly correlated with the prognosis of patients with OC and also involved in N^6^-methyladenosine (m^6^A) regulation. However, its influence on OC progression and the underlying mechanism is still not well demonstrated. Here, we found that UBA6-AS1 directly associated with UBA6 mRNA and inhibited its decay. Further mechanism investigation revealed that UBA6-AS1 increased the m^6^A methylation of UBA6 mRNA via recruiting RNA binding motif protein 15 (RBM15). Insulin like growth factor 2 mRNA binding protein 1 (IGF2BP1) was identified as the m^6^A reader protein of UBA6-AS1-RBM15-mediated m^6^A modification of UBA6 mRNA, which enhanced the stability of UBA6 mRNA. Functionally, UBA6-AS1 suppressed the proliferation, migration and invasion of OC cells via UBA6. Moreover, UBA6-AS1 positively correlated with UBA6 expression in OC tissues. Downregulation of UBA6-AS1 or UBA6 expression indicated poor. Collectively, we have identified a tumor-suppressive lncRNA that regulates its target mRNA via a m^6^A mechanism, highlighting the role that lncRNAs can play in OC progression.

## Introduction

Ovarian cancer (OC) is the seventh most common cancer in women and the main cause of cancer-related death worldwide [1]. The improvement of novel treatments for OC patients has been made in recent years [2–4]. However, with lack of specific clinical signs or symptoms and effective or sensitive clinical detection methods in the early stage, 70% of patients with OC are diagnosed at a middle or advance stage, which leads a high mortality rate of OC. The five-year survival rate of OC patients is below 45% [5]. Therefore, it is essential to uncover the molecular mechanisms underlying OC initiation and progression, which will be great helpful to identify novel effective biomarkers for the diagnosis and treatment of OC.

N^6^-methyladenosine (m^6^A) is the most common RNA modification throughout the transcriptome, regulating fundamental aspects of RNA metabolism. The m^6^A modification can be catalyzed by methyltransferases (Methyltransferase 3 (METTL3), Methyltransferase 14 (METTL14), KIAA1429 and WT1 associated protein (WTAP)), or removed by demethylases (FTO alpha-ketoglutarate dependent dioxygenase (FTO) and alkB homolog 5 (ALKBH5)), which are termed m^6^A ‘writers’ and ‘erasers’, respectively. m^6^A reader proteins are responsible for selective recognition and binding m^6^A-modified RNA, modulating the splicing, decay, translocation, translation, and mature processes [6]. Given that deregulated m^6^A modification results in dysregulation of gene expression related to cell differentiation, proliferation, motility, and invasiveness, m^6^A is indeed involved in tumor initiation and progression [7]. For example, KIAA1429-induced m^6^A promoted the translation of c-MYC, BCL2, and Phosphatase and tensin homolog (PTEN) mRNAs in the human acute myelocytic leukemia (AML) cells, suppressing the differentiation and apoptosis of AML cells [8]. In OC, KIAA1429 and METTL3 is associated with the prognosis of OC patients [9,10]. METTL3 promotes OC growth and invasion through the regulation of AXL receptor tyrosine kinase (AXL) translation and epithelial to mesenchymal transition (EMT) [9].

RETRACTED

Long noncoding RNAs (lncRNAs) are larger than 200 nucleotides in length and do not have a protein-coding function. Abnormal expression of lncRNAs has been observed in human disease and cancer, which participates in the regulation of gene expression at the transcriptional, posttranscriptional and posttranslational level [11–14]. These lncRNAs regulate the malignant behaviors of cancer cells, such as metabolism, proliferation, metastasis, drug resistance angiogenesis [15–17]. Recent reports have indicated that m^6^A methylation is involved in the expression and functions of lncRNAs. For example, METTL14-mediated m^6^A modification enhances the degradation of lncRNA X inactive specific transcript (XIST) via YTH N6-methyladenosine RNA binding protein 2 (YTHDF2), suppressing the proliferation and metastasis in colorectal cancer [18]. LncRNA LNC942 directly recruits METTL14 to stabilize the downstream targets of LNC942 through m^6^A modification [19]. Therefore, lncRNAs can be modified by m^6^A and m^6^A can also modulate their function. A recent study using bioinformatics analysis identified that lncRNA Ubiquitin like modifier activating enzyme 6 antisense RNA 1 (UBA6-AS1) was significantly correlated prognosis and involved in m^6^A regulation for patients with OC [20]. However, to date, the role and mechanism of UBA6-AS1 in OC progression is still not well uncovered.

The present study aims to investigate whether lncRNA UBA6-AS1 plays an important role in modulating OC progression and to reveal the underlying molecular mechanisms via m^6^A modification. Moreover, we evaluated the prognostic value of UBA6-AS1 expression in OC patients.

RETRACTED

## Materials and methods

### Tissue samples collection

Sixty paired OC and corresponding adjacent normal ovary samples were collected from patients who underwent surgery at Hanchuan People’s Hospital between 2014 and 2020. The overall survival was defined as the period between surgery and death or the last follow-up. No radiotherapy or chemotherapy was conducted in these patients before surgery. The diagnosis of OC was confirmed by two experienced pathologists. This study was approved by the Ethics Committee of Hanchuan People’s Hospital. Written informed consent was obtained from all participants enrolled in this study. All the specimens were immediately snap-frozen in liquid nitrogen and stored at −80°C until used.

### Cell culture

The human ovarian cancer cell lines OVCAR3 and SKOV3 were obtained from the Cell Bank of the Chinese Academy of Sciences (Shanghai, China). Cells were cultured in RPMI-1640 medium (Gibco) supplemented with 10% fetal bovine serum (FBS, Biological Industries), 1% penicillin/streptomycin (Gibco) and incubated at 37°C with 5% CO_2_.

### Gene overexpression and knockdown

Full-length UBA6-AS1 sequence was cloned into pLV lentiviral vector. shRNA targeting UBA6-AS1 or UBA6 was inserted into pLV-shRNA lentiviral vector. The target sequence of indicated shRNA was shown as listed: UBA6-AS1 shRNA#1 (KD1): GGGATTGATTACTCCTTGT, UBA6-AS1 shRNA#2 (KD2): TCCCTCTGATTTCAGGCAT, shUBA6: TACAGTCGCAAGCCAAATG. The lentiviral particles were packed in 293 T cells according to the protocol. Cells were infected with indicated lentiviral particles in the presence of polybrene (10 μg/ml). The stable cells were selected by puromycin at a concentration of 5 μg/ml.

### Quantitative real-time PCR (qRT-PCR)

Total RNA was extracted from tissues and cells using the TRIzol Reagent (Invitrogen). 1 μg of total RNA was reverse transcribed using an Evo M-MLV RT Kit with gDNA Clean for qPCR (Accurate Biology). qRT-PCR was performed using a SYBR® Green Premix Pro Taq HS qPCR Kit and the StepOne Plus system (Applied Biosystems). GAPDH was used as the internal control gene. The relative expression levels of indicated genes were calculated using 2^−ΔΔCT^ method. The primer sequences were listed: UBA6-AS1-F: CCGGCTTCTTTACCACTTCTT, UBA6-AS1-R: GGCTGCATTCCTGAGAGATTAG; UBA6-F: TTGGTCCCAGTGTGTAGAATTAG, UBA6-R: AATCGTATGTCCAGAGGGAAAC.

### Western blot

Cells were lysed in RIPA lysis buffer (Beyotime) containing PMSF and then quantified using a bicinchoninic acid (BCA) kit (Thermo Scientific). The equivalent amount of protein samples was separated by 10% sodium dodecyl sulfate polyacrylamide gel electrophoresis (SDS-PAGE) and were transferred to PVDF membranes (Roche). The membranes were blocked and incubated with anti-UBA6 (Abcam), anti-RBM15 (Abcam), anti-IGF2BP1 (Abcam) and anti-GAPDH (Proteintech) overnight, and then incubated with corresponding secondary antibodies. The proteins were detected with Pierce™ ECL Western blotting Substrate.

RETRACTED

### Cell viability assay

Cell viability was measured using the Cell Counting Kit-8 (CCK-8, Dojindo). 2000 cells per well were cultured in 96-well plates with four replicate wells. 10 μl CCK-8 regent was added into each well. After incubation for 1 h, the absorbance at 450 nm was detected using microplate reader (Thermo).

### Migration and invasion assay

Cell migration and invasion was measured on Transwell and Matrigel chamber plates, respectively (8-μm pore size; Corning Costar). Cells were seeded on the Transwell or Matrigel insert membranes, and medium supplemented with 10% FBS was added in the lower chamber. 24 hr later, the upper faces of the filters were abraded with cotton swabs, and cells that had migrated across the filters were fixed in 4% paraformaldehyde and stained with 1% crystal violet.

### Methylated RNA immunoprecipitation (MeRIP)-qRT-PCR

MeRIP assay was carried out according a previous study [21]. Briefly, fragmented mRNA was incubated with m [6]A antibody in 1 ml buffer containing RNase inhibitor (Promega), 50 mM Tris-HCl, 750 mM NaCl and 0.5% (vol/vol) Igepal CA-630 (Sigma Aldrich) for 2 hr. Dynabeads Protein G (Invitrogen) were added to the mixture and incubated for 2 hr with rotation. m^6^A RNA was eluted and purified. m^6^A enrichment of UBA6 mRNA was determined by qRT-PCR.

### RNA immunoprecipitation (RIP)

RIP assay was carried out using the Magna RIP^TM^ RNA-Binding Protein Immunoprecipitation Kit (Millipore) as the manufacturer’s instructions. Briefly, cell lysates were incubated with magnetic beads coated with normal IgG (Millipore), RBM15 (Abcam), METTL5 (Proteintech), IGF2BP1 (Abcam), IGF2BP2 (Abcam), IGF2BP3 (Abcam), METTL3 (Cell Signaling Technology), WTAP (Abcam), YBX1 (Abcam) or GFP (Abcam). The RNA-protein complexes were washed and purified and then subjected to RNA extraction by TRIzol. The UBA6 mRNA enriched by indicated antibody was determined by qRT-PCR. MS2-RIP was performed as previous study described [22].

### RNA pulldown

Biotin-labeled UBA6-AS1 and its antisense RNA were *in vitro* transcribed with the Biotin RNA Labeling Mix (Roche) and T7 RNA polymerase (Roche). After treatment with RNase-free DNase I (Roche), biotinylated RNAs were purified with the RNeasy Mini Kit (Qiagen) and incubated with the indicated cell lysates for 1 h at 4°C. Streptavidin-agarose beads (Invitrogen) were added to each tube and incubated for 1 hr. Finally, the enriched RNA was subjected to qRT-PCR analysis.

RETRACTED

### Statistics

All data are representative of at least three independent experiments. Statistical analysis was performed using SPSS 22.0 software. All data were expressed as the mean ± SD. Student’s t-test was carried out for two group comparisons. One-way analysis of variance ANOVA followed by Dunnett’s post hoc test were used for multiple comparisons. The survival rate was calculated using the Kaplan–Meier method and analyzed by the log-rank test. Pearson’s correlation analysis was applied to analyze the correlation between UBA6-AS1 and UBA6 mRNA levels. P value less than 0.05 was considered statistically significant.

## Results

### UBA6-AS1 associates with UBA6 mRNA and represses its decay

As the antisense RNA of UBA6, we first investigated whether UBA6-AS1 associates with UBA6 and regulates its expression. The result of subcellular fractionation assay demonstrated that UBA6-AS1 was mainly distributed in cytoplasm Figure 1(a), indicating that UBA6-AS1 could regulate target RNAs in a posttranscriptional manner. To detect the interaction between UBA6-AS1 and UBA6 mRNA, the RNA pulldown assay was performed. As shown in Figure 1(b), UBA6 mRNA could be significantly enriched by biotin-labeled UBA6-AS1, but not by the negative control lncRNA HOX transcript antisense RNA (HOTAIR). For further confirmation, we conducted a MS2-RIP followed by qRT-PCR analysis Figure 1(c). It was demonstrated that the UBA6-AS1 RIP was markedly enriched for UBA6 mRNA compared to the empty vector, IgG, or UBA6 binding sites mutated UBA6-AS1 (UBA6-AS1-mut) Figure 1(d). Moreover, as evidenced by the results of qRT-PCR and Western blot experiments, knockdown of UBA6-AS1 significantly decreased both mRNA and protein levels of UBA6, while overexpression of UBA6-AS1 elevated the UBA6 expression Figure 1(e,f). To examine whether UBA6-AS1 regulates the stability of UBA6 mRNA, different clones of OVCAR3 and SKOV3 were treated with actinomycin D, an RNA synthesis inhibitor, and the degradation of UBA6 mRNA was detected at different time points. UBA6-AS1 knockdown significantly accelerated the decay of UBA6 mRNA. Conversely, overexpression of UBA6-AS1 elongated the half-life of UBA6 mRNA Figure 1(g). Taken together, these results suggest that UBA6-AS1 associates with UBA6 mRNA and represses its degradation.

**Figure 1.** UBA6-AS1 associates with UBA6 mRNA and represses its decay a. The cellular location of UBA6-AS1 was detected using subcellular fractionation assay. The U6 and ACTB mRNA was used as nuclear and cytoplasmic internal reference, respectively. b. RNA pull-down assay with biotin-labeled UBA6-AS1 was conducted to detect the interaction between UBA6-AS1 and UBA6 mRNA. LncRNA HOTAIR was used as a negative control. c. The schematic diagram of MS2-RIP experiment. d. MS2-RIP followed by qRT-PCR was performed to detect the association between wild-type or mutant UBA6-AS1 (UBA6-AS1-mut) and UBA6 mRNA. e. The UBA6-AS1 was knocked down and overexpressed in OVCAR3 and SKOV3 cells, and the UBA6-AS1 and UBA6 mRNA levels were tested by qRT-PCR. f. The UBA6-AS1 was knocked down and overexpressed in OVCAR3 and SKOV3 cells, and the UBA6 protein levels were tested by Western blot. g. The OVCAR3 and SKOV3 cells with UBA6-AS1 overexpression or knockdown were treated with actinomycin d, and the UBA6 mRNA levels were tested using qRT-PCR in different time points. *p < 0.05, **p < 0.01, and ***p < 0.001. NC, negative control; KD1, UBA6-AS1 shRNA#1; KD2, UBA6-AS1 shRNA#2; OE, UBA6-AS1 overexpression

RETRACTED

### UBA6-AS1 increases the m^6^A level of UBA6 via recruiting RBM15

LncRNAs are capable to regulate their target RNAs via m^6^A modification [21,23]. UBA6-AS1 is also involved in m^6^A regulation for patients with OC [20]. Hence, we speculated that UBA6-AS1 may regulate the UBA6 expression via m^6^A modification. To validate this, MeRIP assay was carried out. The m^6^A level of UBA6 mRNA was significantly decreased by depletion of UBA6-AS1 Figure 2(a). Conversely, overexpression of UBA6-AS1 obviously increased the m^6^A methylation of UBA6 mRNA compared to control cells Figure 2(a). According to the bioinformatics analysis from a previous study, UBA6-AS1 was correlated with m^6^A ‘writers’, Methyltransferase 5 (METTL5) and RNA binding motif protein 15 (RBM15) [20]. We performed an RIP assay and found that RBM15, but not METTL5, could associated with UBA6-AS1 Figure 2(b). Furthermore, knockdown of UBA6-AS1 significantly attenuated the association between RBM15 and UBA6 mRNA, whereas this interaction was enhanced by UBA6-AS1 overexpression Figure 2(c).

**Figure 2.** UBA6-AS1 increases the m^6^A level of UBA6 via recruiting RBM15 a. The m^6^A levels of UBA6 mRNA in OVCAR3 and SKOV3 cells with UBA6-AS1 overexpression or knockdown was examined using MeRIP followed by pRT-PCR. b. RIP assay using negative control IgG, RBM15 or METTL5 antibody was conducted to detect the amount of UBA6-AS1 associated with RBM15 or METTL5. c. RIP analysis of RBM5-associated UBA6 mRNA in OVCAR3 and SKOV3 cells with UBA6-AS1 overexpression or knockdown. d. siRNA targeting RBM15 was transfected into OVCAR3 and SKOV3 cells with UBA6-AS1 overexpression, and the RBM15 and UBA6 mRNA levels were assessed using qRT-PCR. e. siRNA targeting RBM15 was transfected into OVCAR3 and SKOV3 cells with UBA6-AS1 overexpression, and the RBM15 and UBA6 protein levels were assessed using Western blot. f. siRNA targeting RBM15 was transfected into OVCAR3 and SKOV3 cells with UBA6-AS1 overexpression, and the loss of UBA6 mRNA was assessed using qRT-PCR. g. RIP analysis of METTL3- or WTAP-associated UBA6 mRNA in OVCAR3 and SKOV3 cells with UBA6-AS1 overexpression or knockdown. *p < 0.05, **p < 0.01, and ***p < 0.001. NC, negative control; KD1, UBA6-AS1 shRNA#1; KD2, UBA6-AS1 shRNA#2; OE, UBA6-AS1 overexpression

Then, we detected whether UBA6-AS1 modulates the UBA6 expression via RBM15. UBA6-AS1-overexpressed cells were transfected with RBM15 siRNA. Then, the mRNA and protein expression of UBA6 was tested using qRT-PCR and Western blot, respectively. We found that silence of RBM15 abolished the UBA6-AS1-mediated upregulation of UBA6 Figure 2(d,e). Consistently, the stability of UBA6 mRNA was reversed by RBM15 knockdown Figure 2(f).

RETRACTED

RBM15 was identified as a regulator that binds to METTL3 and WTAP and directs these two proteins to m^6^A-modified RNA [24]. Hence, we tested whether UBA6-AS1 could affect the interaction of UBA6 mRNA with METTL3 and WTAP. It was shown by RIP assay that the association between METTL3 or WTAP and UBA6 mRNA was attenuated after transfection of UBA6-AS1 shRNA, but enhanced by ectopic expressing UBA6-AS1 in OC cells Figure 2(g). Collectively, these findings suggest that UBA6-AS1 elevates the m^6^A level of UBA6 via recruiting RBM15.

### IGF2BP1 is involved in the UBA6-AS1-RBM15-mediated stability of UBA6 mRNA

Then, we validated which m^6^A reader protein is involved in the UBA6-AS1-RBM15-mediated stability of UBA6 mRNA. Insulin-like growth factor 2 mRNA binding proteins (IGF2BPs) recognize and bind with the m^6^A-modified mRNAs, thus enhancing their stability [6]. We performed RIP assays using IGF2BPs antibody and found that only IGF2BP1 associated with UBA6 mRNA, which was repressed by UBA6-AS1 knockdown, but promoted by UBA6-AS1 overexpression Figure 3(a,b). Furthermore, downregulation of IGF2BP1 abolished the UBA6-AS1-induced increase of UBA6 expression and stability Figure 3(c-e).

**Figure 3.** IGF2BP1 is involved in the UBA6-AS1-RBM15-mediated stability of UBA6 mRNA a. RIP assay using negative control or IGF2BPs antibody was carried out to test the association of UBA6 mRNA with IGF2BPs. b. RIP analysis of IGF2BP1-associated UBA6 mRNA in OVCAR3 and SKOV3 cells with UBA6-AS1 overexpression or knockdown. c. siRNA targeting IGF2BP1 was transfected into OVCAR3 and SKOV3 cells with UBA6-AS1 overexpression, and the IGF2BP1 and UBA6 mRNA levels were assessed using qRT-PCR. d. siRNA targeting IGF2BP1 was transfected into OVCAR3 and SKOV3 cells with UBA6-AS1 overexpression, and the IGF2BP1 and UBA6 protein levels were assessed using Western blot. e. siRNA targeting IGF2BP1 was transfected into OVCAR3 and SKOV3 cells with UBA6-AS1 overexpression, and the loss of UBA6 mRNA was assessed using qRT-PCR. f. RIP analysis of YBX1-associated UBA6 mRNA in OVCAR3 and SKOV3 cells with UBA6-AS1 overexpression or knockdown. *p < 0.05, **p < 0.01, and ***p < 0.001. NC, negative control; KD1, UBA6-AS1 shRNA#1; KD2, UBA6-AS1 shRNA#2; OE, UBA6-AS1 overexpression

Oncoprotein Y-box binding protein 1 (YBX1) interacts with IGF2BP1, which is critical for IGF2BP1 in stabilizing m^6^A-tagged RNA [25]. For this reason, we examined whether UBA6-AS1 affects the binding of UBA6 mRNA with YBX1. As evidenced by RIP assay, the interaction between YBX1 and UBA6 mRNA was weakened by deletion of UBA6-AS1 expression, but promoted by ectopic expressing UBA6-AS1 in OC cells Figure 3(f). Together, these data suggest that UBA6-AS1-RBM15 increases UBA6 expression via m^6^A reader protein IGF2BP1.

RETRACTED

### UBA6-AS1 exerts tumor-suppressive roles via UBA6

Then, the functional role of UBA6-AS1 was investigated in OC cells. Cell proliferation detection using CCK-8 assay showed that overexpression of UBA6-AS1 significantly repressed the proliferation ability of both OVCAR3 and SKOV3 cells, which was rescued by transfection of UBA6 shRNA Figure 4(a,b). Furthermore, the cell migration and invasion were tested using transwell assays. Overexpression of UBA6-AS1 significantly attenuated the motility and invasiveness of OC cells, while knockdown of UBA6 abolished this suppression Figure 4(c-d). These data suggest that UBA6-AS1 inhibits the malignant behaviors of OC cells via UBA6.

**Figure 4.** UBA6-AS1 exerts tumor-suppressive roles via UBA6 a. UBA6 was knocked down in OVCAR3 and SKOV3 cells with UBA6-AS1 overexpression by shRNA against UBA6, and the UBA6 expression was examined by qRT-PCR. b. UBA6 was knocked down in OVCAR3 and SKOV3 cells with UBA6-AS1 overexpression, and then the cell proliferation was assessed by CCK-8 assay. c. UBA6 was knocked down in OVCAR3 and SKOV3 cells with UBA6-AS1 overexpression, and then the cell migration was assessed by transwell assay. The represent images and statistical result were shown. d. UBA6 was knocked down in OVCAR3 and SKOV3 cells with UBA6-AS1 overexpression, and then the cell invasion was assessed by Matrigel-coated transwell assay. The represent images and statistical result were shown. e. qRT-PCR analysis of the UBA6-AS1 levels in 60 pairs of OC and matched normal ovary tissue samples. f. qRT-PCR analysis of the UBA6 mRNA levels in 60 pairs of OC and matched normal ovary tissue samples. g. The Pearson’s correlation analysis between UBA6-AS1 and UBA6 mRNA levels in OC tissues. h. Kaplan-Meier survival analysis of overall survival in OC patients based on UBA6-AS1 expression. The median of UBA6-AS1 expression in OC tissues was used as cutoff. i. Kaplan-Meier survival analysis of overall survival in OC patients based on UBA6 mRNA expression. The median of UBA6 mRNA expression in OC tissues was used as cutoff. *p < 0.05, **p < 0.01, and ***p < 0.001. NC, negative control; KD1, UBA6-AS1 shRNA#1; KD2, UBA6-AS1 shRNA#2; OE, UBA6-AS1 overexpression

Finally, the clinical significance of UBA6-AS1 and UBA6 expression was investigated. The UBA6-AS1 and UBA6 mRNA in 60 pairs of OC and matched normal ovary tissues were examined using qRT-PCR. It was shown that both UBA6-AS1 and UBA6 mRNA was markedly downregulated in OC tissues compared to normal tissues Figure 4(e-f). Additionally, correlation analysis revealed that UBA6-AS1 positively correlated with UBA6 mRNA in OC tissues Figure 4(g). Furthermore, we assessed the prognostic values of UBA6-AS1 and UBA6 expression using Kaplan–Meier method and found that patients with higher UBA6-AS1 or UBA6 expression always had longer median overall survival as compared with those with lower UBA6-AS1 or UBA6 expression Figure 4(h,i). These data suggest a prognostic value of UBA6-AS1 and UBA6 expression for OC patients.

RETRACTED

## Discussion

In recent years, some lncRNAs have been identified as important regulators of gene expression, such as lncRNA Differentiation antagonizing non-protein coding RNA (DANCR) and Pro-transition associated RNA (PTAR), which play important roles in modulating OC initiation and progression [26,27]. Bioinformatics analysis identified that UBA6-AS1 was significantly correlated prognosis of OC patients [20]. Consistently, we found that UBA6-AS1 expression was significantly decreased in OC tissues. OC patients with low UBA6-AS1 expression had shorter overall survival than those with high expression of UBA6-AS1. Functional experiments demonstrated that overexpression of UBA6-AS1 not only repressed OC cell proliferation, but also inhibited the motility and invasiveness of OC cells. Thus, our findings indicated that lncRNA UBA6-AS1 acts as a tumor suppressor in OC and may be used as a potential prognostic indicator for OC.

To the best of our knowledge, our research was the first to reveal the mechanism of UBA6-AS1 in OC. Here, our results showed a tumor-suppressive function of UBA6-AS1 in OC cells. Cytoplasmic lncRNAs can post-transcriptionally regulate gene expression. For example, lncRNA PTAR acts as a competing endogenous RNA (ceRNA) of miR-101 and decreases its expression and activity, thus upregulating Zinc finger E-box binding homeobox 1 (ZEB1) expression in OC [28]. LncRNA Metastasis associated lung adenocarcinoma transcript 1 (MALAT1) directly binds to SRY-box transcription factor 2 (Sox2) mRNA and represses its degradation in gastric cancer cells [29]. Nevertheless, the mechanism by which lncRNA affects its interacting mRNA remains largely unknown. Our present study showed that UBA6-AS1 mainly located in cytoplasm, associated with UBA6 mRNA and inhibited its decay. Consistent with our findings, antisense lncRNAs have been found to stabilize target mRNAs. For example, lncRNA MACC1-AS1 stabilizes MACC1 mRNA in gastric cancer [30]. Moreover, lncRNA PDCD4-AS1 stabilizes PDCD4 RNA by forming RNA duplex and controls the interaction between PDCD4 RNA and HuR [31]. Recently, the lncRNA-regulated m^6^A modification gains massive attention. For instance, long non-coding RNA antisense to FOXM1 (FOXM1-AS) promotes the interaction of ALKBH5 with Forkhead box M1 (FOXM1) nascent transcripts, leading to enhanced FOXM1 expression [21]. DNA methylation-deregulated and RNA m^6^A reader-cooperating lncRNA (DMDRMR) binds IGF2BP3 to stabilize target mRNAs, including Cyclin dependent kinase 4 (CDK4), Collagen type VI alpha 1 chain (COL6A1), Laminin subunit alpha 5 (LAMA5), and Fibronectin 1 (FN1), by specifically enhancing IGF2BP3 activity on them in a m^6^A-dependent manner [23]. Here, we demonstrated that UBA6-AS1 recruited ‘writer’ RBM15 to UBA6 mRNA, and then enhanced the binding of METTL3 and WTAP with UBA6 mRNA, resulting in increased m^6^A methylation of UBA6 mRNA. Subsequently, IGF2BP1 and YBX1 recognized and bound the m^6^A-tagged UBA6 mRNA to inhibit its decay. Recent studies also revealed that lncRNAs are involved in other RNA modification. NSUN2 increases 5-methylcytosine (m^5^C) modification of lncRNA H19, which enhances the interaction between H19 and oncoprotein G3BP1 [32]. Additionally, lncRNA FOXC2-AS1 facilitates FOXC2 mRNA stability via elevating its m^5^C level [33]. These findings highlight a close relationship between lncRNAs and RNA modification.

RETRACTED

UBA6 is a ubiquitin activating enzyme and acts as a tumor suppressor in breast cancer. Depletion of UBA6 promotes cell cycle progression and invasion by stabilization of ezrin, Cell division cycle 42 (CDC42) and CUGBP Elav-like family member 1 (CUGBP1) [34]. We found that UBA6 expression was downregulated in OC tissues. Decreased UBA6 expression also indicated poor clinical outcome of OC patients. UBA6-AS1 was positively correlated with UBA6 expression in OC tissues. Moreover, UBA6-AS exerted suppressive effects via UBA6. All these findings suggested that UBA6 was a bona fide downstream of UBA6-AS1. However, there are some limitations in our research. Firstly, we did not identify the exact m^6^A sites of UBA6 mRNA. Secondly, *in vivo* study will further confirm our *in vitro* findings. Thirdly, the binding area between UBA6-AS1 and RBM15 needs further investigation.

## Conclusions

Taken together, these results demonstrate that UBA6-AS1 inhibits the malignant phenotypes via stabilizing UBA6 mRNA in a m^6^A-dependent manner (Figure 5), and UBA6-AS1 may be a novel prognostic indicator for OC patients.

**Figure 5.** The schematic diagram of proposed mechanism of UBA6-AS1 in OC cells

## Data Availability

All data supporting the findings of this study are available within the paper.
